The article "Study of OH• Radicals in Human Serum Blood of Healthy Individuals and Those with Pathological Schizophrenia" was published in 2011. Journal: Int J Mol Sci.

# Study of OH^•^ Radicals in Human Serum Blood of Healthy Individuals and Those with Pathological Schizophrenia

**DOI:** 10.3390/ijms12010401

**Published:** 2011-01-14

**Authors:** Elena I. Korotkova, Bashkim Misini, Elena V. Dorozhko, Mariya V. Bukkel, Evgeniy V. Plotnikov, Wolfgang Linert

**Affiliations:** 1 Tomsk Polytechnic University, Lenin av., 30, 634050, Tomsk, Russia; 2 Institute of Applied Synthetic Chemistry, Vienna University of Technology, Getreidemarkt 9/163AC A–1060 Vienna, Austria; E-Mail: wlinert@mail.zserv.tuwien.ac.at (W.L.)

**Keywords:** human serum blood, fluorimetry, hydroxyl radicals, terephthalic acid, schizophrenia

## Abstract

The human body is constantly under attack from free radicals that occur as part of normal cell metabolism, and by exposure to environmental factors such as UV light, cigarette smoke, environmental pollutants and gamma radiation. The resulting “Reactive Oxygen Species” (ROS) circulate freely in the body with access to all organs and tissues, which can have serious repercussions throughout the body. The body possesses a number of mechanisms both to control the production of ROS and to cope with free radicals in order to limit or repair damage to tissues. Overproduction of ROS or insufficient defense mechanisms leads to a dangerous disbalance in the organism. Thereby several pathomechanisms implicated in over 100 human diseases, e.g., cardiovascular disease, cancer, diabetes mellitus, physiological disease, aging, *etc.*, can be induced. Thus, a detailed investigation on the quantity of oxygen radicals, such as hydroxyl radicals (OH^•^) in human serum blood, and its possible correlation with antioxidant therapy effects, is highly topical. The subject of this study was the influence of schizophrenia on the amount of OH^•^ in human serum blood. The radicals were detected by fluorimetry, using terephthalic acid as a chemical trap. For all experiments the serum blood of healthy people was used as a control group.

## 1. Introduction

Mental disorders like drug abuse, depression, schizophrenia, *etc.* are increasingly affecting societies worldwide. Clinical schizophrenia is connected with a number of vegetative, psychological and biochemical processes in a human organism [1]. One of the current focuses in this field of research is the investigation of the relation of various malfunctions caused by mental disorders like schizophrenia [1,2].

Schizophrenia affects men and women equally. It occurs at similar rates in all ethnic groups around the world. Symptoms such as hallucinations and delusions usually start between ages 16 and 30. It can be difficult to diagnose schizophrenia in teens. This is because the first signs can include a change of friends, a drop in grades, sleep problems, and irritability—behaviors that are common among teenagers [3].

Schizophrenia is caused by several factors. Scientists have long known that schizophrenia runs in families. The illness occurs in 1 percent of the general population, but it occurs in 10 percent of people who have a first-degree relative with the disorder, such as a parent, brother, or sister. Other recent studies suggest that schizophrenia may result in part when a certain gene, that is key to making important brain chemicals, malfunctions. This problem may affect the part of the brain involved in developing higher functioning skills. In addition, it probably takes more than genes to cause the disorder. Scientists think interactions between genes and the environment are necessary for schizophrenia to develop. Many environmental factors may be involved, such as exposure to viruses or malnutrition before birth, problems during birth, and other not yet known psychosocial factors [4,5].

Scientists think that an imbalance in the complex, interrelated chemical reactions of the brain involving the neurotransmitters dopamine and glutamate, and possibly others, plays a role in schizophrenia. Neurotransmitters are substances that allow brain cells to communicate with each other [6].

Five sub-classifications of schizophrenia are known [7]:

- Paranoid type: Where delusions and hallucinations are present but thought disorder, disorganized behavior, and affective flattening are absent.
- Disorganized type: Named hebephrenic schizophrenia. Where thought disorder and flat affect are present together.
- Catatonic type: The subject may be almost immobile or exhibit agitated, purposeless movement. Symptoms can include catatonic stupor and waxy flexibility.
- Undifferentiated type: Psychotic symptoms are present but the criteria for paranoid, disorganized, or catatonic types have not been met.
- Residual type: Where positive symptoms are present at a low intensity only.
- Post-schizophrenic depression: A depressive episode arising in the aftermath of a schizophrenic illness where some low-level schizophrenic symptoms may still be present.
- Simple schizophrenia: Insidious and progressive development of prominent negative symptoms with no history of psychotic episodes.

Scientists have learned a lot about schizophrenia, but more research is needed to help explain how it develops. The ROS play major role in development of schizophrenia.

This work will develop better treatment to help people with schizophrenia achieve their full potential.

It is well known that mental illnesses significantly affect the antioxidant protective system of an organism which might lead to oxidative damage caused by a rapid growth of free oxygen radicals [8–15]. Thus a detailed research of oxygen radical’s quantity in human serum blood under pathological conditions (schizophrenia) and the investigation of its possible correlation with antioxidant therapy efficiency is highly prospective.

Detection of OH^•^ radicals in human serum blood under pathological conditions of schizophrenia was carried out by fluorimetry, whereby terephthalic acid (TA) was used as a chemical trap.

It is known that reactive oxygen species (ROS) are involved in diseases like cancer, atherosclerosis, hepatocirrhosis, psychotropic diseases, *etc.* Direct detection of ROS is practically impossible because of their extreme reactivity and very short lifetime. This led to the development of chemical traps to facilitate their quantitative detection [16], where the potential of ROS to oxidize a chemical trap is defined as Fenton activity. The most commonly used procedure is based on the hydroxylation of salicylic acid, which is based on the chemical reaction shown in Scheme 1:

However, some authors [17,18] have questioned its validity. Accurate quantitative estimation of ROS formation could be achieved only if all three hydroxylation products are considered. However, species I, as it is produced only in small amounts is usually neglected in the analysis. Even so, under the assumption of a constant ratio of the hydroxylation products, it should still be possible to obtain reliable ROS quantification by taking two or even only one derivative. Recent experiments in our laboratories, however, confirmed by several results from the literature, have shown that there is time dependence and, moreover, strong influence of chemical environment on the product ratio, affecting even *in vitro* results. Several additional problems arise under *in vivo* conditions. Species II is also produced enzymatically, leaving only species III available for detection as a simple ROS product. As the ratio between species III and species II varies from 5:1 to 1:1 the resulting quantization error is far from being negligible. Moreover, species III is quite unstable and, in common with the other species, quickly metabolized. Furthermore, salicylic acid itself is biologically active and could influence inflammatory processes associated with oxidative stress, thus directly affecting the results.

W. Freinbichler and Prof. W. Linert *et al.* [19] developed a new fluorimetric method for detection of ROS, using terephthalic acid (H_2_TA) as a chemical trap. Formation of ROS like OH^•^ radicals can be detected by the ROS producing model reaction like the Fenton reaction [19] (Equation 1), whereby the non-fluorescent H_2_TA is hydroxylated to the excellent fluorophor TA-OH.

$${\text{Fe}}^{2+}+{\text{H}}_{2}{\text{O}}_{2}\to {\text{Fe}}^{3+}+2{\text{OH}}^{\cdot }$$

Hydroxylation of terephthalic acid occurs as presented in Scheme 2:

A big advantage of this system is that, apart from some minor fragmentation products, which occur in all aromatic hydroxylation processes, the symmetry of the molecule leads to only one hydroxylated product which in contrast to the (quasi) non fluorescent TA^2−^ gives brilliant fluorescence.

Based on this system, we were able to develop the method of OH^•^ radical detection in human serum blood in patients with pathological schizophrenia.

## 2. Materials and Methods

To determine the number of OH^•^ radicals in human serum blood a RF-5301pc Spectrofluorophotometer Shimadzu (Germany) was used. The pH values of the solutions were monitored using a Theta’90, M-150 pH-meter (Czechia).

### 2. 1. Preparation of serum sample

During this study serum blood of 50 healthy males aged from 20 to 30 (without pathology) and 10 male patients aged from 23 to 42 with paranoid type of schizophrenia (clinical form) treated in psychiatric hospital was used. It is known schizophrenia affects men and women equally [3]. In this work only the male patients were chosen for investigation. During the experiment blood had been tested three times for 10 days. Before the experiments blood centrifuging had been carried out for 10 minutes at 1500 rpm [20].

### 2. 2. Detection of OH^•^ radical’s concentration in serum blood by fluorimetry

#### 2.2.1. Preparation of standard solutions

A standard solution of sodium salt of terephthalic acid (sodium terephthalate Na_2_TA) with the concentration of 1·10^−2^ mol/L was prepared by dissolving 0.166 g of terephthalic acid H_2_TA (Technical University of Vienna, Austria) in 100 mL of NaOH (0.01 mol/L). A standard solution of Mohr’s salt (NH_4_)_2_Fe (II) (SO4)_2_·(6H_2_O) (Merk) with the concentration of 2 × 10^−3^ mol/L was prepared by dissolving 0.024 g in 50 mL of distilled water. A standard solution of H_2_O_2_ with the concentration of 1 × 10^−3^ mol/L was prepared from a 30% solution (Sigma-Aldrich) by taking 0.05 mL of that solution into 20 mL of distilled water. The exact concentration of H_2_O_2_ was determined by titrating it with KMnO4.

As a supporting solution phosphate buffer (0.025 mol/L, pH = 6.86 (equimolar mixture of Na_2_PO_4_ and KH_2_PO_4_) with 2% KCl (for 100 mL of a standard solution of buffer of 2 g of KCl)) was used.

#### 2.2.2. Detection of OH^•^ radicals in Fenton system

Reactive oxygen species (ROS), that exist either as free or bound hydroxyl radicals or Fe(IV) oxo species, selectively hydroxylate the non-fluorescent TA to the brilliant fluorophor 2-hydroxy-terephthalic acid (TA-OH).

To detect the fluorescence signal of TA-OH in a Fenton system, the following solutions were added in a particular order into a cell of 10 mL: —2 mL of standard solution of terephthalate (1·10^−2^ mol/L); —0.03 mL of standard solution of Mohr’s salt (2·10^−3^ mol/L); —0.03 mL of standard solution of hydrogen peroxide (1·10^−3^ mol/L); —2 mL of supporting solution of phosphate buffer at pH = 6.86.

The remaining volume was adjusted to the mark using distilled water (V = 6.4 mL). The mixture was incubated at room temperature for 6 minutes.

To investigate the quantity of hydroxyl radicals in serum blood, 2 mL of terephthalate (1·10^−2^ mol/L) standard solution, 2 mL of supporting solution and different volumes of serum from 0.1 to 0.5 mL were added into the 10 mL cell. The remaining volume of the reaction mixture was adjusted to the mark using distilled water.

Within this work OH^•^ radicals in serum blood of 10 healthy males and 10 male patients with schizophrenia were detected by fluorimetry, using terephthalic acid. Detailed emission spectra have been obtained for an excitation wavelength of 315 nm at a pH of 6.86.

A Fenton system (Equation 1) was used to generate OH^•^ radicals and the signal of TA-OH was measured fluorimetrically.

## 3. Results and Discussion

In Figure 1 the emission spectrum of the reaction product of terephthalic acid with OH^•^ radicals (TA-OH) at λ = 327 nm (see Scheme 2) is presented. These data are in excellent agreement with those in [15]. In Figure 2, the dependence on the signal strength of TA-OH on hydrogen peroxide concentration (mmol/L) is presented. A linear dependence in the range of H_2_O_2_ concentrations from 0.1mmol/L to 0.5 mmol/L was observed (Figure 2). For each concentration the three samples of hydrogen peroxide were used to obtain each measure.

For the quantitative detection of OH^•^ radicals in human serum blood in patients with pathological schizophrenia the detected fluorescence spectrum was identical to that of TA-OH with λemission_max_ = 327 nm (Figure 3) for excitation wavelength of 315 nm at a pH of 6. 86. It was concluded that TA-OH was the only fluorescing species under these conditions. The received signal increased with addition of serum blood (Figure 3).

The results lead to the assumption that natural components of human serum blood contain a system able to generate active OH^•^ radicals, which can be defined using fluorimetry. In turn, the controlling the maintenance of active OH^•^ radicals in human serum blood will reveal the increase or decrease of ROS levels in the blood that can be key to understanding important biochemical processes developed in an organism with pathological symptoms of mental illnesses. In Figure 4 the dependence on the peak intensity of TA-OH fluorescence on the volume of added human serum blood, taken from healthy males and patients with pathological schizophrenia with an identical duration of the illness, is presented. All examples show a similar linear behavior. For each volume the three samples of human serum blood were used to obtain each measure.

Thus, in this work, a quantitative detection of active OH^•^ radicals in serum blood of healthy people and patients with pathological schizophrenia by fluorimetry was carried out. Table 1 presents the results obtained from 10 healthy patients and with pathological scizophrenia.

As one can see from Table 1, concentrations of OH^•^ radicals in serum blood of healthy patients are considerably lower than in serum blood of people with pathological schizophrenia. Probably, the high content of OH^•^ radicals in the serum of patients in comparison to healthy people may be due to lipid peroxidation of biomembranes of cells during the development of the pathology, resulting in increased secretion of OH^•^ radicals in the blood, which is in excellent agreement with the literature [19]. It is known [21,22] that the concentration of peroxide radical in the blood of healthy people is in region of 200–400 μmol/L, measured photometrically by immune diagnostic assay.

Thus, the quantity of OH^•^ radicals in human serum blood under physiological and pathological conditions of schizophrenia was determined by fluorimetry. It was revealed that in serum blood of healthy people, there are less OH^•^ radicals generated than in the blood of people suffering from schizophrenia. The results clearly show that the presented techniques could be very helpful for clinical laboratories for the purpose of operational control for the content of active oxygen radicals in human blood, which eventually could lead to a better understanding of important biochemical processes taking place in the body with pathological symptoms of mental illnesses. The present technique is very simple; therefore, its implementation would be easy for routine use.

## Figures and Tables

**Figure 1:** Fluorescence TA-OH in Fenton system at λ = 327 nm.

**Figure 2:** Dependence on peak intensity of fluorescence TA-OH on hydrogen peroxide concentration in the solution. N = 3.

**Figure 3:** The fluorescence spectrum of TA-OH in human serum blood in patients with pathological schizophrenia at λ= 327 hm. **----**0.1 mL of serum blood; ----0.2 mL of serum blood; ----0.25 mL of serum blood.

**Figure 4:** Dependence on the peak intensity of TA-OH fluorescence on the volume of human serum blood of healthy males and patients with pathological schizophrenia. ---serum blood of healthy male, ---serum blood of patient No1, ---serum blood of patient No2,---serum blood of patient No3. N = 3.

**Scheme 1:** Hydroxylation of Salicylic acid.

**Scheme 2:** Hydroxylation of terephthalic acid due to radical oxidation.

**Table 1:** Concentrations of OH^•^ radicals in serum blood of healthy people and patients with pathological schizophrenia.

The code of the patient	Concentration of OH^•^ radicals in serum blood of healthy people, μmol/L	Concentration of OH^•^ radicals in serum blood of patients with schizophrenia, μmol/L
1	400 ± 2.02	520 ± 2.53
2	350 ± 1.31	510 ± 2.16
3	390 ± 1.21	550 ± 4.61
4	410 ± 3.04	580 ± 2.53
5	310 ± 3.52	420 ± 2.72
6	290 ± 1.91	430 ± 1.91
7	340 ± 3.13	450 ± 2.84
8	270 ± 2.42	380 ± 4.03
9	300 ± 2.82	520 ± 4.51
10	320 ± 4.13	560 ± 3.23
